# A Changing Landscape in Castration-Resistant Prostate Cancer Treatment

**DOI:** 10.3389/fendo.2012.00085

**Published:** 2012-07-18

**Authors:** A. Felici, M. S. Pino, Paolo Carlini

**Affiliations:** ^1^Department of Medical Oncology, Regina Elena National Cancer InstituteRome, Italy; ^2^Medical Oncology Unit, Department of Oncology, Azienda Sanitaria FirenzeFlorence, Italy

**Keywords:** prostate cancer, castration-resistance, sipuleucel-T, cabazitaxel, abiraterone, denosumab

## Abstract

Prostate cancer (PC) is the leading cause of cancer and the second leading cause of cancer-death among men in the Western world. About 10–20% of men with PC present with metastatic disease at diagnosis, while 20–30% of patients diagnosed with localized disease will eventually develop metastases. Although most respond to initial androgen-deprivation therapy (ADT), progression to castration-resistant PC (CRPC) is universal. In 2004 the docetaxel/prednisone regimen was approved for the management of patients with metastatic CRPC, becoming the standard first-line therapy. Recent advances have now led to an unprecedented number of new drug approvals within the past years, providing many new treatment options for patients with metastatic CRPC. Four new drugs have received U.S. Food and Drug Administration (FDA)-approval in 2010 and 2011: sipuleucel-T, an immunotherapeutic agent; cabazitaxel, a novel microtubule inhibitor; abiraterone acetate, a new androgen biosynthesis inhibitor; and denosumab, a bone-targeting agent. The data supporting the approval of each of these agents are described in this review, as are current approaches in the treatment of metastatic CRPC and ongoing clinical trials of novel treatments and strategies.

## Introduction

Prostate cancer (PC) is the leading cause of cancer and the second leading cause of cancer-death among men in the Western world (Siegel et al., 2012). For early stage PC definitive primary treatment with surgery and radiation is often curative. Unfortunately, about 10–20% of men with PC present with metastatic disease at diagnosis, while 20–30% of patients diagnosed with localized disease will eventually develop metastases. Androgen-deprivation therapy (ADT) is the mainstay of initial therapy in these patients, and involves the use of luteinizing hormone-releasing hormone (LHRH) drugs (agonists or antagonists; chemical castration) or orchiectomy (surgical castration), consistently resulting in a 90–95% reduction in circulating levels of testosterone. However, nearly all patients will develop progressive disease, despite castrate levels of androgens (testosterone level < 50 ng/mL), namely castration-resistant prostate cancer (CRPC), after a median duration of response of 18–24 months (Hamberg et al., 2008; Sternberg, 2008). Although secondary hormonal manipulations (including antiandrogens, and androgen-suppressing agents, such as estrogens and ketoconazole) can benefit a subset of men with metastatic CRPC, this benefit is usually short-lived.

Prior to 2004, there was no treatment proven to improve survival for men with metastatic CRPC. Mitoxantrone in combination with prednisone was explicitly developed, and approved as a palliative agent with no increase in overall survival (OS; Tannock et al., 1996; Kantoff et al., 1999). In 2004, the docetaxel/prednisone regimen was approved for the management of patients with metastatic CRPC. This approval was based on two landmark phase III trials (TAX 327 and SWOG 9916), which demonstrated a survival benefit of approximately 2 months for docetaxel in combination with either prednisone or estramustine (Petrylak et al., 2004; Tannock et al., 2004). In the TAX 327 trial, patients with metastatic CRPC were randomized to receive two different schedules of docetaxel (weekly or every 3 weeks) plus prednisone, or mitoxantrone with prednisone. A significant survival benefit favoring docetaxel every 3 weeks compared to mitoxantrone [hazard ratio (HR) for death, 0.76, 95% CI, 0.62–0.94; *p* = 0.009] was observed, together with an improved quality of life, lower levels of cancer-induced bone pain, decreased serum levels of PSA and superior response rates (Tannock et al., 2004). In 2008, an updated survival analysis of this study showed that the significant survival benefit with docetaxel every 3 weeks compared with mitoxantrone persisted even with extended follow-up, with a median OS of 19.2 and 16.3 months (*p* = 0.004), respectively (Berthold et al., 2008). In the SWOG 9916 phase III trial docetaxel in combination with estramustine was compared with mitoxantrone in combination with prednisone, with a survival advantage in the group treated with docetaxel (17.5 vs. 15.6 months; HR for death, 0.80; 95% CI, 0.67–0.97; *p* = 0.02; Petrylak et al., 2004).

While the absolute gain in median survival of docetaxel-based chemotherapy was statistically and clinically significant, improving its efficacy and prolonging the relatively short duration of its benefit have continued to be matter of studies. Moreover, until 2010, there were no treatment options conferring a survival benefit for patients with docetaxel-refractory CRPC, although mitoxantrone was often employed in this setting for its palliative effects on bone pain. Within the past year, several agents with different mechanisms of action have demonstrated efficacy, and in 2012 therapeutic options for patients with metastatic CRPC include four new agents approved by the U.S. Food and Drug Administration (FDA) in 2010 and 2011. These new agents are an immunotherapeutic product (sipuleucel-T), for the treatment of asymptomatic or minimally symptomatic metastatic CRPC patients; a novel taxane, cabazitaxel, which showed a survival advantage over mitoxantrone in docetaxel-pretreated patients; an androgen synthesis inhibitor, abiraterone acetate, which was also reported to improve survival when evaluated against placebo in docetaxel-pretreated patients; and a bone-targeting agent (denosumab; Table 1).

**Table 1:** **New therapies in CRPC**.

Trial	Agent	Control arm	CRPC population	Benefit
TAX327 (Tannock et al., 2004; Berthold et al., 2008)	Docetaxel	Mitoxantrone + prednisone	Chemo-naïve	Survival benefit (19.2 vs. 16.3)
IMPACT (Kantoff et al., 2010a)	Sipuleucel-T	Placebo	Chemo-naïve (>80%)	Survival benefit (25.8 vs. 21.7)
TROPIC (de Bono et al., 2010)	Cabazitaxel	Mitoxantrone + prednisone	Docetaxel-refractory	Survival benefit (15.1 vs. 12.7)
COU-AA-301 (de Bono et al., 2011)	Abiraterone	Placebo + prednisone	Docetaxel-refractory	Survival benefit (14.8 vs. 10.9)
ALSYMPCA (Parker et al., 2012b)	Radium-223	Placebo	Docetaxel-refractory	Survival benefit (14.9 vs. 11.3)

## Immune-Based Therapy

Several approaches that attempt to treat PC by activating an immune response against malignant cells, while overcoming tumor-induced tolerance and avoiding autoimmune reactions have been undertaken. Indeed, the slow-growing nature of the disease may allow a stimulated immune system the necessary time to generate an antitumor response and to overcome immunosuppressive factors. Several tissue-specific proteins, recently identified by both proteomic and microarray studies, may serve as tumor antigens, such as PSA and prostate acid phosphatase (PAP). Preclinical data have demonstrated the feasibility of eliciting an antitumor immune response against PC, especially when active immunotherapy is combined with immune checkpoint blockade, androgen ablation, or radiotherapy (Coffey and Isaacs, 1981; Rhodes et al., 2002; Wang et al., 2005; Drake et al., 2006; Taylor et al., 2006; Arlen et al., 2009; Di Lorenzo et al., 2010; Drake, 2010; Gulley and Drake, 2011).

There are currently multiple immunological strategies in clinical development for PC. Those that have generated the most interest in recent years include the sipuleucel-T (Provenge®) autologous PAP-loaded dendritic cell product, the GVAX allogeneic recombinant whole cell platform, the Prostvac-VF poxviral vector vaccine, a PAP-encoding DNA vaccine, and approaches that inhibit the immune checkpoints CTLA-4 (cytotoxic T-lymphocyte-associated antigen-4; Arlen et al., 2009; Di Lorenzo et al., 2010; Drake, 2010; Gulley and Drake, 2011).

### Antigen-presenting cell vaccines

The FDA approved sipuleucel-T (APC8015, Provenge®; Dendreon Corporation, Seattle, WA, USA) on April 29, 2010 to treat asymptomatic or minimally symptomatic metastatic CRPC. Shortly afterward, sipuleucel-T was added to the compendium of cancer treatments published by the National Comprehensive Cancer Network (NCCN) as a “category 1” (highest recommendation) treatment for CRPC.

Sipuleucel-T is a first-in-class active cellular immunotherapy product that is manufactured by collecting peripheral blood mononuclear cells by leukopheresis. The cells are then exposed, for 36–44 h, to a recombinant fusion protein (PA2024) consisting of granulocyte macrophage colony-stimulating factor (GM-CSF), which is an established immune response-enhancing agent, and PAP, which is expressed by cancerous and non-cancerous prostatic cells. Activated dendritic cells, expressing PA2024 as antigens on their cell surface, are infused back into the patient and are then capable of sensitizing naïve T-cells to develop reactivity toward PA2024, specifically the PAP peptide portion. The final product also contains a variable number of T-cells, B-cells, natural killer cells, as well as other cells. The entire process (including leukapheresis and *in vitro* stimulation) is repeated three times, once every 2 weeks (Higano et al., 2010).

Two randomized, placebo-controlled, phase III trials, with time to progression (TTP) as the primary end point, were initially carried out (D9901 and D9902A; Small et al., 2006). Neither of the studies meet the primary end point although median OS was improved by 4 months over placebo in the first study (25.9 vs. 21.4 months, *p* = 0.01). A *post hoc* pooled analysis of these two trials in a total of 225 asymptomatic metastatic CRPC patients, of which 147 randomized to sipuleucel-T and 78 to placebo, confirmed the survival advantage with a 33% reduction in the risk of death compared to placebo (HR 1.50; 95% CI, 1.10–2.05; *p* = 0.011; Higano et al., 2009). Nevertheless, because OS was not the primary endpoint in either trial, the FDA recommended further data in support of the efficacy claim. A larger, double blind, placebo-controlled, multicenter phase III study, the IMPACT (IMmunotherapy for Prostate AdenoCarcinoma Treatment) was subsequently conducted in 512 patients with asymptomatic or minimally symptomatic metastatic CRPC with OS as the primary endpoint (Kantoff et al., 2010a). Patients were randomly assigned in a 2:1 ratio to either the treatment (341 patients) or the placebo arm (171 patients). In the final analysis, sipuleucel-T arm demonstrated a 22.5% reduction in the risk of death (HR 0.775; 95% CI, 0.61–0.98; *p* = 0.03) compared to the placebo arm, together with a 4.1 months improvement in median survival (25.8 vs. 21.7 months). Furthermore, the sipuleucel-T group showed a 3-year survival of 32.1% compared to 23.0% in the placebo group, indicating that a small proportion of patients significantly benefit from treatment. Interestingly, neither PSA response rate, nor objective radiological responses were observed. Results from immunologic testing confirmed the drug activity on a biological level, with a higher titer of antibodies against PA2024 in patients receiving sipuleucel-T and who had a prolonged survival (*p* < 0.001). In these studies the most common adverse events were chills, fatigue, fever, dyspnea, back pain, nausea, joint ache, headache, local-injection reaction, most of which were mild and transient, occurring within 1 day of infusion and resolving within 24–48 h. The most serious adverse events reported were acute infusion reactions, and cerebrovascular events, the latter occurring at a very low rate, and without statistically significant difference between arms.

The enigmatic advantage in OS, despite the unmeet traditional end-points such as progression-free survival (PFS) or PSA response, is an uncommon finding. The most plausible explanation is the inadequacy of our current clinical metrics of progression. Immune responses to vaccines require time to develop (minimum 12 weeks), which can translate into an even longer period to demonstrate a benefit, and the lack of differences in progression could result from delayed antitumor responses occurring after PSA or radiologic progression (Wolchok et al., 2009). It is understandable that in clinical practice, ignoring a continually raising PSA and added risk of progression while waiting for an immune response, will have obvious ethical implications. That is why for patients with tumor-related symptoms who need rapid tumor shrinkage to provide palliation, or patients with rapidly progressive disease, upfront chemotherapy should be preferred. Despite FDA approval, many questions still remain as to how sipuleucel-T should be used. After treatment with sipuleucel-T, many patients presumably will move onto other treatment, many of which involving the use of immunosuppressive steroids, but the appropriate timing for this is unclear.

At present, there are a number of clinical trials underway involving sipuleucel-T. In the neoadjuvant setting, currently ongoing but not recruiting, the NeoACT (NEOadjuvant Active Cellular ImmunoTherapy) phase II trial will assess the immune response within prostate tissue following neoadjuvant treatment with sipuleucel-T in patients scheduled for radical prostatectomy. Furthermore, following radical prostatectomy subjects will be randomized to receive either a booster of sipuleucel-T or no further treatment.

### Viral vector vaccines

Viruses are a convenient vehicle for vaccine delivery, due to large genomes that allow for insertion of multiple genes for tumor-associated antigens (TTAs), co-stimulatory molecules, and cytokines; the ability to cause an inflammatory response at the injection site with migration of APCs to the site, or to directly infect the APCs allowing for better antigen processing; and most of all are relatively easy and inexpensive to produce as compared with immunotherapy products based on autologous antigen-presenting cells. Vaccine therapies are generally well tolerated, with the most common adverse effects being infusion reactions or reversible flu-like symptoms within the first few days after treatment. Yet, host-induced antibodies can neutralize the vector and limit its efficacy with repeated use. Recently, a prime-boost strategy has been developed, whereby replication-competent vaccinia virus primes the immune system, and then a replication-defective avipox virus, such as fowlpox, which is not associated with significant neutralizing antibodies, boosts it (Acres and Bonnefoy, 2008; Amato et al., 2008; Dreicer et al., 2009; Liu, 2010).

PROSTVAC®-VF (BN ImmunoTherapeutics, Inc., Mountain View, CA, USA) is a pox viral vaccine consisting of fowlpox and vaccinia vectors engineered to express the human *PSA* gene, and a triad of co-stimulatory molecules, known as TRICOM^TM^ (intercellular adhesion molecule-1 or ICAM-1, T-lymphocyte activation antigen CD80 or B7.1, and lymphocyte function-associated antigen 3 or LFA-3). In a randomized, double blind, placebo-controlled phase II trial of PROSTVAC-VF (one priming dose, then 6 boosts over 24 weeks) in metastatic, chemotherapy-naïve, CRPC no significant difference in PFS, primary endpoint, was observed. However, a striking 8.5 months survival advantage was seen in the treatment arm 3 years post-study as compared to the control arm (25.1 vs. 16.6 months, HR 0.56; 95% CI 0.37–0.85; *p* = 0.0061; Kantoff et al., 2010b). Mirroring early finding with sipuleucel-T, there was no difference in the serum PSA responses, or the PSA antibody titers between treatment groups, despite PSA being the targeted tumor antigen, with no evidence of specific anti tumor effects. The Eastern Cooperative Oncology Group recently activated a phase II randomized study (ECOG 1809) of docetaxel with or without PROSTVAC-VF as first-line therapy for men with metastatic CRPC. This study will address relevant sequencing questions and may determine whether chemotherapy is additive to immunotherapy.

### Immunostimulatory agents

A spontaneous antitumor immune response can be induced by a non-specific stimulation. Ipilimumab is a human monoclonal antibody that binds to cytotoxic T-lymphocyte antigen-4 (CTLA-4), a negative regulator of T-cell-mediated antitumor immune responses, already approved for treating chemotherapy-refractory metastatic melanoma patients (Hodi et al., 2010). Anti-CTLA-4 monoclonal antibodies binding to CTLA-4 on T-cell prolongs T-cell activation, restores T-cell proliferation, and thus amplifies T-cell-mediated immunity, which enhances the patient’s capacity to mount an antitumor immune response. In metastatic CRPC patients, phase I data showed some evidence of clinical responses, both as single agent as well as in combination with radiation therapy (Beer et al., 2008). In a phase I dose-escalating study ipilimumab in combination with GM-CSF showed PSA as well as radiological responses. A correlation between higher ipilimumab doses and effectiveness was also shown by an increased number of circulating activated CD8^+^ cells detected by flow-cytometry (Fong et al., 2009). Two phase III trials are currently recruiting patients: one comparing ipilimumab vs. placebo following a low-dose of radiation to a bone lesion, in order to release tumor antigens from dying tumor cells, in metastatic docetaxel-pretreated CRPC patients (NCT00861614), and the other comparing the efficacy of ipilimumab vs. placebo in asymptomatic or minimally symptomatic patients with metastatic chemotherapy-naïve CRPC (NCT01057810).

## Cytotoxic Chemotherapy

In 2004, docetaxel with prednisone was approved for the use in CRCP patients on the basis of a 2.5 months survival advantage over mitoxantrone and prednisone (Petrylak et al., 2004; Tannock et al., 2004). In addition docetaxel improved global and pain-based quality of life measures when compared with mitoxantrone. Until recently, there were no chemotherapeutic options approved for the treatment of CRPC after progression on docetaxel. Today a new agent has received FDA approval, and new chemotherapies are in advanced clinical development.

### Cabazitaxel

Cabazitaxel (Jevtana®, Sanofi-Aventis, U.S.; Bridgewater, NJ, USA) is a novel semi-synthetic taxane, and as such stabilizes microtubules thereby inhibiting their disassembly and inducing cell cycle arrest. In contrast to other taxanes has a low affinity for the adenosine triphosphate-dependent drug efflux pump P-glycoprotein 1, which can be responsible for docetaxel resistance. In 2010, a phase III trial, the TROPIC trial, randomized 755 patients with metastatic CRPC, after docetaxel failure, between cabazitaxel plus prednisone and mitoxantrone plus prednisone (de Bono et al., 2010). A 2.4-months survival advantage was reported in the cabazitaxel arm (15.1 vs. 12.7 months), corresponding to a 30% reduction in the risk of death (HR: 0.70; 95% CI, 0.59–0.83; *p* < 0.0001). Secondary end-points such as PFS (2.8 vs. 1.4 months; *p* = 0.0002), response rate (14.4 vs. 4.4%; *p* = 0.0005), and median TTP by tumor assessment (8.8 vs. 5.4 months; *p* < 0.0001) also favored cabazitaxel. Comparing the adverse event profile of these agents, the most frequent toxicity in the cabazitaxel group was neutropenia of grade 3 or higher (82 vs. 58%). The incidence of febrile neutropenia was also higher with cabazitaxel (8 vs. 1%), as was diarrhea (6 vs. <1%). Treatment-related deaths, primarily for infectious complications and renal failure, were more frequent with cabazitaxel. The FDA approved cabazitaxel in combination with prednisone in June 2010. Special attention should be given to prevent febrile neutropenia and infections with primary prophylactic use of G-CSF in high-risk patients. It is currently ongoing a phase III randomized trial (FIRSTANA) in chemo-naïve patients with CRPC, which compared two different doses of cabazitaxel, plus prednisone vs. docetaxel plus prednisone. Primary objective is OS (NCT01308567).

## Hormonal Therapy

Androgens are the primary regulators of PC cell growth and proliferation, and indeed ADT nearly always leads to a PSA response. However, despite the initial response to first-line hormonal therapy, the median duration of response is 18–24 months, and the development of CRPC is inevitable (Hamberg et al., 2008; Sternberg, 2008). It is well known that CRPC involves in most cases the reactivation of the androgen receptor (AR) in the absence of gonadal testosterone. Continued AR activation occurs likely from one or more of several mechanisms including: amplification or overexpression of the *AR* gene, mutations of the *AR* gene, changes in the levels of AR cofactors, increased expression of enzymes involved in androgen synthesis, ligand-independent activation of AR, and enhanced intracellular conversion of adrenal androgens to testosterone and dihydrotestosterone (Dayyani et al., 2011). Clinical PC progression reflects a gradual shift from endocrine sources of androgens (especially from the testes and adrenal glands) to paracrine, autocrine, and intracrine sources within the tumor microenvironment (Stanbrough et al., 2006; Mizokami et al., 2009). Hence, CRPC tumors are not uniformly hormone-refractory and may remain sensitive to therapy directed against the AR axis. Indeed several new classes of AR-targeting agents are now in clinical development, including CYP17 inhibitors that suppress the steroidogenesis, such as abiraterone acetate, and potent AR antagonists, such as MDV3100.

### Abiraterone

Abiraterone acetate (Zytiga®, Janssen-Cilag International NV) is an orally administered inhibitor of 17 α-hydroxylase and C_17,20_-lyase referred to as the CYP17 complex, a member of the cytochrome P450 family. CYP17 is a microsomal enzyme and catalyzes 2 reactions, the 17 α-hydroxylation of pregnenolone and progesterone to 17 αOH-pregnenolone and 17α OH-progesterone, respectively, and the subsequent C_17,20_-lyase reaction to form the corresponding 17-keto androgens, namely dehydroepiandrosterone and androstenedione, which are precursors of all other androgens, including testosterone. Inhibition of the CYP17 complex leads to accumulation of upstream mineral corticoids and reduction of downstream steroids including testosterone and estradiol. In fact, abiraterone side effects are dependant on mineralocorticoid excess, and include hypokalemia, hypertension, peripheral edema, and headaches (Reid et al., 2008). These adverse events are in most cases controlled by administration of corticosteroids or aldosterone antagonist. Abiraterone treatment has been shown to suppress testosterone levels, with reduction in PSA level, regression of radiological lesions, and improvement in symptoms in phase I and II studies conducted in docetaxel-naïve and docetaxel-pretreated patients (Attard et al., 2008, 2009a; Danila et al., 2010; Reid et al., 2010; Ryan et al., 2010). These results led to two randomized placebo-controlled phase III trials testing the efficacy of abiraterone in improving survival in patients with metastatic CRPC. A randomized, double blind, placebo-controlled trial (COU-AA-301) compared abiraterone plus prednisone with placebo plus prednisone in 1,195 docetaxel-pretreated patients with CRCP (de Bono et al., 2011). Based on a 4 months improvement in OS found at the interim analysis (14.8 vs. 10.9 months; HR 0.65; 95% CI 0.54–0.77; *p* < 0.0001), as well as significant improvements in PFS (5.6 vs. 3.6 months; *p* < 0.001) and overall response rate (38 vs. 10%; *p* < 0.001), abiraterone was FDA approved in April 2011 for metastatic CRPC patients that previously received docetaxel-based chemotherapy. A second phase III trial (COU-AA-302) comparing abiraterone plus prednisone vs. placebo plus prednisone in patients with metastatic CRPC who are chemotherapy-naïve has recently completed accrual. Primary end-points of the study are OS and PFS (NCT00887198). The final results are due for reporting in the next months.

### MDV3100

MDV3100 is a potent novel small AR antagonist that blocks testosterone binding to AR, and prevents the nuclear translocation and DNA binding of the ligand-AR complex. Unlike bicalutamide, MDV3100 does not possess agonist activity when AR is overexpressed (Attard et al., 2009b; Tran et al., 2009). In a phase I/II study of 140 patients to determine the maximum tolerated dose, safety, pharmacokinetics, and antitumor activity of MDV3100, an antitumor effect was seen in both chemotherapy-naïve and docetaxel-pretreated patients (Scher et al., 2010). Fifty-six percent of patients had 50% or greater PSA decline, 22% of the patients with measurable disease had a partial response, and 56% of the patients with bone disease had a stable disease; the median TTP for all patients was of 47 weeks. Based on these encouraging results, a phase III trial (AFFIRM) was conducted to compare MDV3100 vs. placebo in metastatic CRPC patients who had previously received docetaxel-based chemotherapy. Results are pending (NCT00974311). A second phase III trial (PREVAIL) evaluating the impact of MDV3100 vs. placebo in chemotherapy-naïve patients with metastatic CRCP, with OS and PFS as co-primary end-points, is currently recruiting (NCT01212991).

## Bone-Targeting Agents

Patients with CRPC have an increased risk of skeletal-related events (SREs), including fracture, progressive bone pain, spinal cord compression, due to reduced bone mineral density from castration, frequent glucocorticoid use, other than disease process. More than 80–90% of patients with metastatic CRPC will develop bone metastases, resulting in substantial morbidity and a significant detrimental effect on quality of life. In a double blind, phase III trial in men with metastatic CRPC the intravenous bisphosphonate zoledronic acid (4 mg intravenously every 3 weeks) showed a significant reduction in the rate of SREs as compared to placebo (44.2 vs. 33.2%; *p* = 0.021), with a delay in the time to a first SRE (Saad et al., 2002). Patients who were treated with zoledronic acid also had significantly decreased in urinary markers of bone resorption. An analysis of the long-term efficacy of zoledronic acid in 122 patients from the original study confirmed a significant trend in improved outcomes, with an ongoing risk of experiencing a SRE reduced by 36% (Saad et al., 2004).

Denosumab (XGEVA®, Amgen, Thousand Oaks, CA, USA), is a fully human monoclonal antibody against receptor activator of nuclear factor-kappa B (RANK) ligand, a key protein secreted by stromal cells and osteoblast in response to growth factors released by tumor cells, which promotes osteoclast activation by binding the RANK-receptor on their surface. The ligand-receptor interaction causes the activation of survival and proliferation pathways in osteoclasts that trigger bone resorption (Li et al., 2000; Mundy et al., 2001). Denosumab (60 mg) was first evaluated in a double blind phase III trial of ADT-related bone loss compared with placebo administered every 6 months (Smith et al., 2009). After 2 years, the lumbar spine bone mineral density increased by 5.6% in the denosumab arm, whereas it decreases by 1.0% in the placebo arm (*p* < 0.001), with similar increases in the bone mineral density of the total hip, femoral hip, and distal third of the radius. These improvements led to a significant decreased 3 year incidence of new vertebral fractures among patients in the denosumab arm (*p* = 0.006). In a second trial denosumab (120 mg subcutaneously every 4 weeks) was compared with zoledronic acid (4 mg endovenously every 4 weeks), in 1,904 men with bone metastases from CRPC (Fizazi et al., 2011). In this study, denosumab significantly delayed the time to first on-study SRE (HR 0.82; 95% CI, 0.71–0.95; *p* = 0.008), with a median time of first on-study SRE of 20.7 months compared to 17.1 months in patients receiving zoledronic acid, a difference of 3.6 months, and an overall risk reduction of 18%. Overall survival (HR 1.03; 95% CI, 0.91–1.17; *p* = 0.65) and time to cancer progression (HR 1.06; 95% CI, 0.95–1.18; *p* = 0.30) were similar between the two treatment arms. Adverse event rates were similar, with primarily fevers, constipation, and joint pain; rates of hypocalcemia were higher in the denosumab arm (13 vs 6%; *p* < 0.0001), with osteonecrosis of the jaw being more frequent in the experimental arm (*p* = 0.09). The FDA approved in November 2010 denosumab for the prevention of SREs in men with metastatic CRPC and bone metastases. Phase III studies evaluating the ability of these agents to delay the development of bone metastases are ongoing.

Alpharadin (radium-223 chloride) is a first-in-class, highly targeted α-emitting radiopharmaceutical under clinical evaluation for CRPC patients with bone metastases. By carrying microscopic amounts of radium-223, which acts as a calcium mimic, alpharadin delivers high energy, short range irradiation that induces double-stranded DNA breaks with lower penetration to surrounding tissues, compared with the β-emitting radiopharmaceuticals samarium-153 and strontium-89. In the phase III ALSYMPCA (ALpharadin in SYMptomatic Prostate CAncer) alpharadin has shown both delayed time to first SRE and an unprecedented OS benefit (Parker et al., 2012a; Sartor et al., 2012). The ALSYMPCA study was stopped early after a pre-planned efficacy interim analysis, on the basis of achieving a statistically significant improvement in OS (median OS 14.0 vs. 11.2 months, HR = 0.699; *p* = 0.0022). Updated data showed that alpharadin improved OS by 44% (HR = 0.695; *p* = 0.00007), resulting in a 30.5% reduction in the risk of death compared to placebo (Parker et al. 2012b). The median OS benefit with alpharadin was 3.6 months in this updated analysis (14.9 months in patients given alpharadin vs. 11.3 months with placebo). Alpharadin has been granted Fast Track designation by the FDA.

## Conclusions

The availability of multiple new treatments in patients with metastatic CRPC is the current challenge for the clinicians, now facing the choice of the right treatment at the right time (Figure 1). In our view, sipuleucel-T would be the most appropriate treatment for naïve patients with asymptomatic to minimally symptomatic bone- or lymph node-metastatic CRPC, which do not require immediate treatment with chemotherapy. Indeed, symptomatic patients would be probably better served with chemotherapy as sipuleucel-T administration leads to almost no response, as well as TTP is not affected. It can be anticipated that lack of availability, complexity of administration, approval of the center by the manufacturer, and cost issues will probably limit clinical utilization of sipuleucel-T in the near future. In patients with symptomatic disease or visceral metastases, or in those who have a rapidly progressive disease, chemotherapy should be administered, and docetaxel with prednisone is the preferred first choice. In docetaxel-pretreated patients, phase III trials support the use of cabazitaxel or abiraterone, preferred in frail men, each given with prednisone. Docetaxel retreatment may also be appropriate, especially in patients with a good initial response to docetaxel and subsequent discontinuation for reasons other than disease progression. In addition to the above approaches, the use of bone health-promoting agents such as denosumab or zoledronate should be strongly considered for men with bone metastatic disease to prevent pathological fractures, spinal cord compression or the need for radiation or surgery for skeletal complications.

**Figure 1:** **The current treatment paradigm of CRPC**.

## Conflict of Interest Statement

The authors declare that the research was conducted in the absence of any commercial or financial relationships that could be construed as a potential conflict of interest.
